# A Small Sample Recognition Model for Poisonous and Edible Mushrooms based on Graph Convolutional Neural Network

**DOI:** 10.1155/2022/2276318

**Published:** 2022-08-12

**Authors:** Li Zhu, Xin Pan, Xinpeng Wang, Fu Haito

**Affiliations:** College of Information Technology, Jilin Agriculture University, ChangChun 130118, Jilin, China

## Abstract

The automatic identification of disease types of edible mushroom crops and poisonous crops is of great significance for improving crop yield and quality. Based on the graph convolutional neural network theory, this paper constructs a graph convolutional network model for the identification of poisonous crops and edible fungi. By constructing 6 graph convolutional networks with different depths, the model uses the training mechanism of graph convolutional networks to analyze the results of disease identification and completes the automatic extraction of the disease characteristics of the poisonous crops by overfitting problem. During the simulation, firstly, the relevant PlantVillage dataset is used to obtain the pretrained model, and the parameters are adjusted to fit the dataset. The network framework is trained and parameterized with prior knowledge learned from large datasets and finally synthesized by training multiple neural network models and using direct averaging and weighting to synthesize their predictions. The experimental results show that the graph convolutional neural network model that integrates multi-scale category relationships and dense links can use dense connection technology to improve the representation ability and generalization ability of the model, and the accuracy rate generally increases by 1%–10%. The average recognition rate is about 91%, which greatly promotes the ability to identify the diseases of poisonous crops.

## 1. Introduction

Digital image processing is usually used for the identification of poisonous crop diseases and poisonous crop diseases, and the image segmentation process is usually performed. When the field light changes or the background is complex, the effect of image segmentation will be affected, thereby reducing the subsequent recognition rate [1–4]. In addition, this method requires the extraction of a large number of features, and the high computational complexity will reduce the recognition efficiency. The zero-sample image recognition of edible mushrooms aims to solve the problem of identifying target categories without labeling data. Most of the current zero-shot image recognition methods for edible mushrooms try to map the visual features of the image and the semantic features of the category into a shared embedding space and then use the nearest neighbor search algorithm in the shared embedding space to determine the category label of the image [5–7].

Because the categories contained in the training set and the test set are different, and the manifold structure of the image feature space and the semantic feature space is inconsistent, this type of method often has problems such as projection domain drift, mapping bias, and pivot points. To alleviate the above problems, this paper studies the problem of zero-sample image recognition of edible mushrooms with the help of category hierarchy relationship, graph convolutional neural network, and reversible generative model [8–11]. Therefore, combining the image characteristics of edible mushroom samples, and integrating the graph convolutional network method into the ATR of edible mushroom samples is an important research direction for intelligent interpretation of edible mushroom samples. Carrying out the research on the target recognition method of edible mushroom samples based on a graph convolutional network is helpful to enhance the target perception and information processing capabilities of the edible mushroom sample system, which has a profound impact on national defense security construction and national economic development [12].

Aiming at the problem of the decline of the network recognition ability under the small sample of edible tannin, the convolutional neural network fine-tuning method for target recognition of edible tannin samples was studied. Aiming at the problems of the current generation model-based zero-sample image recognition method for edible mushrooms, the lack of diversity of generated data, and insufficient model expression ability, this paper adopts a new reversible generative model CNFG based on conditional regular flow to solve the problem of edible mushroom zero and sample image recognition problem. To better take control measures against the disease of poisonous crops according to the degree of disease, a method for identifying the disease level of crop leaves based on an improved convolutional neural network is proposed. First, it may preprocess the selected leaf image data, including illumination processing, image segmentation, pixel extraction of disease spots, etc., and then divide the preprocessed diseased leaves into different grades according to the severity. In terms of algorithm improvement, the focal loss function and the optimization algorithm were used to optimize the model and improve the recognition accuracy, reaching 95.61%.

## 2. Related Work

Scholars from various countries have conducted in-depth research on the classic three-level processing mechanism of ATR, and have achieved fruitful results. However, the research on ATR of edible mushroom samples based on graph convolutional networks is still in the stage of continuous exploration and innovation, and there are many problems to be solved urgently [13–15]. For example, there are many types of graph convolutional networks, but their structural design lacks standardized theoretical guidance, which largely depends on the designer's subjective experience. If a single network is used, it may lead to poor recognition performance due to wrong structure selection; graph convolutional networks and strong learning adaptability of the network and the large-scale training sample set are inseparable. The training ability of the graph convolutional network requires repeated iterative operations, resulting in long network optimization and low target recognition efficiency. The research and solution to the above problems are of great significance for constructing an ATR system for edible mushroom samples with higher recognition efficiency and stronger recognition ability, and for promoting the development of image interpretation of edible mushroom samples towards a higher level of intelligence [16].

The more visual description proposed by Shen [17] is the core idea of the early stage of zero-sample image recognition of edible tannin. Traditional image recognition methods usually map input images directly to class labels and perform end-to-end learning. The drawbacks of this end-to-end learning approach emerge when encountering images of categories that do not appear in the training set. Early zero-sample image recognition methods for edible mushrooms based on attribute classifiers were to learn more fine-grained attribute features in the image and then determine the category of objects according to the attribute features. Barhoom [18] designs a corresponding matching algorithm for various image information (such as color, texture, shape, gradient, etc.), and then obtains targeted image features (such as scale-invariant feature transformation SIFT, directional gradient histogram HOG, and color histogram HSV, etc. This method of acquiring image features not only relies too much on expert knowledge but also has low generalization of the acquired features, which is not conducive to extending to other image processing tasks. Early zero-sample image recognition of edible mushrooms all used such image features, resulting in a generally low recognition rate for images of unknown categories in early models. With the maturity of artificial neural network technology, Mahelawi [19] found that the image features extracted using the convolutional neural network model have achieved good results in the spatial structure of “intraclass” distance and “interclass” distance, and have very good results, and generalization performance is very high. Therefore, the current zero-sample image recognition methods for edible tannins generally use convolutional neural networks to extract image features. Yan [20] proposed a CVAE model, which takes the attribute feature vector of the category as the condition, directly generates the image feature data of the unknown category with the help of conditional variational auto-encoding, and finally uses the support vector machine SVM as the image feature classifier. Ma [21] also pointed out that the data generated by conditional variational auto-encoding lacks multimodality and cannot well express the data distribution of real data. Therefore, experts make further improvements to the CVAE model, by introducing a feedback-driven learning algorithm, which inversely maps the output of the decoder to the category attribute features, thereby making the generated data more discriminative. Different from existing methods that represent the prototype of a category as a vector point in a high-dimensional space, scholars use the latent spatial distribution of a specific category to represent the prototype of the category and then use these latent spatial distributions as prior knowledge to train variational autoencoders [22–26].

## 3. Graph Convolutional Neural Network Small Sample Recognition

### 3.1. Graph Convolutional Network Solution Set

In the test phase of the graph convolutional network, the visual feature *x* of the test image is first extracted by the deep neural network, and then according to different feature space mapping schemes, the similarity with the category prototype is selected in different shared embedding spaces, and then the similarity of the image is determined. For example, in the first mapping method that chooses the semantic space as the shared embedding space, the test image feature *x* will be passed through the function.

(1) $$\begin{array}{c} \left\{\begin{array}{c} \sum \frac{w\left(x,t\right)}{w\left(x\right)}=\sum \frac{u\left(x,t\right)}{u\left(x\right)}-\frac{u\left(t\right)}{t},\\ \sum \frac{x\left(t\right)}{t}=\sum \frac{u\left(t\right)}{t}-\frac{u\left(x\right)}{w\left(x\right)}. \end{array}\right) \end{array}$$

Since transductive learning can utilize some additional information in the test set, such as data distribution and manifold space structure, the performance of transductive learning is usually better than that of inductive learning. The two learning paradigms mentioned above also exist in the field of zero-sample image recognition of edible mushrooms, and there are also two methods for predicting category labels, namely transductive prediction and inductive prediction.

(2) $$\begin{array}{c} \frac{\text{sig mod}\left(x,y\right)}{\text{exp}\left(x\right)\text{exp}\left(t\right)}=\frac{1-\text{exp}\left(x,t\right)}{\text{exp}\left(x\right)-\text{exp}\left(t\right)}. \end{array}$$

If the adjacency matrix A is multiplied directly by the node vector *X*, that is, AX, it is equivalent to adding all the neighbor node vectors of a node in Table 1, and replacing them with the value of the current node.

Since the edible mushroom samples are imaged according to the electromagnetic scattering characteristics of the ground objects, the edible mushroom samples are highly sensitive to the azimuth angle of the target, but the actual training samples are often difficult to cover all the azimuth angles of the target.

(3) $$\begin{array}{c} \left\{\begin{array}{c} u\left(n,n-1\right)*u\left(n,1\right)=1,\\ v\left(1-n\right)\left(n,n-1\right)*x\left(n,1-n\right)=1. \end{array}\right) \end{array}$$

Therefore, the training samples can be augmented by attitude synthesis to compensate for the reduction of target information caused by the lack of azimuth angle, and reduce the sensitivity of the network to the target attitude. The fully connected layer contains a large number of trainable parameters, which increases the difficulty of network training, and the network depth has an important impact on the representation ability of deep neural networks.

### 3.2. Network Small Sample Gradient

The first 8 gradient feature maps of the small sample C31 take the four adjacent feature maps in S21 as input respectively, the 9th to 15th feature maps take the six nonadjacent feature maps in S21 as the input, and the last feature map connect with all feature maps in S21. According to the connection method shown in nodes 3–3, C31 contains a total of 4034 trainable parameters, which is 2254 less than the nonsparse convolution.

(4) $$\begin{array}{c} e\left(x,n\right)=\left\{\begin{array}{c} 1-u\left(n,n-1\right),\\ 1-\frac{1-x}{u\left(n,1\right)}. \end{array}\right) \end{array}$$

To further illustrate the superiority of the improved model, the prediction results of each category of the final improved model are compared with the results of each category predicted by the original VGG16 model. The test accuracy of the VGG16 model ranges from 92.27% to 99.35%, and the final improved model test accuracy is between 95.00% and 99.70%. Due to the complex shooting background of the category anthracnose leaf blight and the 3rd category leaf rust disease, the noise interference is relatively large, and it is relatively difficult to identify.

There is a serious data imbalance problem in the ImageNet test set, that is, the number of samples contained in each category in Figure 1 varies greatly. In addition, due to the low generalization performance of the current edible mushroom zero-sample image recognition on ultra large-scale datasets, only using the top-1 accuracy rate cannot effectively evaluate the performance of the model. As suggested, the paper uses the category-based average top *k* accuracy as the evaluation metric.

(5) Re rspern,m=maxm−hLiLk−1+k,n−hLiLk−1+k.

The convolution features of inception block1, inception block2, and inception block3 are extracted and fused using a multi-feature fusion method. It is verified through experiments that the use of multi-layer fusion features to train the recognition model can effectively supplement the lack of single-layer networks. The pooling layer is generally after the convolution layer, and based on the principle of local correlation, the feature map of the lower layer of the network is down-sampled, the data features are integrated, and the complexity of network training is reduced to a certain extent.

### 3.3. Graph Convolutional Network Weight Decay

Graph convolutional network weights are connected in a local-aware manner. Taking an input image of 1000 × 1000 pixels as an example, assuming that the first network layer has 10,000 neurons, for a fully connected network, this would result in 10 connections and the same order of magnitude of trainable parameters. If the local perception method is adopted, assuming that the size of the receptive field is 10, the corresponding number of connections is 10, which is reduced to 1/10,000 of the original number of connections. Therefore, local awareness significantly reduces the number of parameters of the graph convolutional network, which will greatly help to improve the network training rate.

(6) $$\begin{array}{c} 1-\frac{\partial w\left(x,y,z\right)}{\partial w\left(z\right)\partial y\;\partial x}=\left\{\begin{array}{c} \frac{\partial w\left(x,y,z\right)}{\partial w\left(x\right)\partial y\;\partial z},\\ \frac{\partial w\left(x,y,z\right)}{\partial w\left(y\right)\partial x\;\partial z}. \end{array}\right) \end{array}$$

A shared set of weights is called a convolution kernel or filter, and its output is called a feature map. This weight-sharing convolution method can be understood as using the same filter to extract the same feature in different positions of the image. A convolutional layer usually includes multiple convolution kernels to extract diverse image features. Although DBN solves the training problem of the deep neural networks, the value range of the output of each neuron in the network is limited to [0, 1], and it is not effective to directly use it to model images of real-valued edible mushroom samples. Therefore, this paper will use the graph convolutional network as the basic model for target recognition of edible mushroom samples.

### 3.4. Small Sample Overfitting Distribution

And by training models with different depths of single-layer features in 10 crop disease image datasets, it is found that the network structure is generally the last layer of convolutional features with stronger comprehensive expression ability, and the trained models hold more than those trained with other layer features. However, when the network parameters are not set properly, such as when the learning rate is too large, the ReLU function can easily lead to the “death” of neurons, making the gradient of neurons always 0, and the parameters cannot be updated. The leaky ReLU function avoids the situation that the gradient of Figure 2 is 0 when the input is negative and solves the neuron death phenomenon that exists in the ReLU function.

Severity is one of the most commonly used metrics to measure the extent of disease in plant populations. The ratio of the diseased area in a plant or organ can be expressed as disease severity, such as the total area of the diseased area in leaves of apple scab disease and the ratio to the total area of the entire diseased leaf. The grading method can be used to express the severity, that is, according to a certain standard, the severity of the disease is divided into several grades according to the degree of severity, and each grade can be represented by the percentage of the area of the diseased area or a specified representative value. Therefore, to remove redundant information and reduce computational overhead before feature concatenation, a necessary operation is to perform dimensionality reduction on each feature matrix.

The cascade-equivalent approach can expand the range of the receptive field of the convolution kernel in Figure 3, and at the same time improve the nonlinear representation ability of the network. Two stacked 3 × 3 convolution kernels and one 5 × 5 convolution kernel have the same size of perception range. And, a 5 × 5 convolution kernel contains a total of 5 × 5 + 16 trainable parameters, and two cascaded 3 × 3 convolution kernels contain a total of 3 × 3 + 12 trainable parameters, less than 77.00% of the original parameter. At the same time, the cascade of small convolution kernels increases the number of convolution layers. Correspondingly, the network contains more nonlinear operations, which is beneficial to the abstraction and fitting of complex sample features in the edible mushroom sample image. The basic classification network 2 includes 8 convolutional layers and 3 pooling layers, among which, C32 and C42 two 3 × 3 convolutional layers are concatenated to obtain a 5 × 5 perceptual area. A 3 × 3 convolutional layer is cascaded, equivalent to a 7 × 7 perceptual area.

## 4. Construction of a Small Sample Recognition Model for Toxins and Edible Mushrooms Based on Graph Convolutional Neural Network

### 4.1. Depth Iteration of Graph Convolutional Networks

The zero-sample image recognition method for edible mushrooms based on the graph convolutional network model mainly has four components, which are the image feature extraction module, the class relation graph building module, the graph convolutional neural network building module, and the loss function calculation module. Among them, the image feature extraction technology is very mature, and the paper directly uses the existing relatively mature deep convolutional neural network for image feature extraction. The experimental results are as shown, as the network layer increases, the crop disease recognition rate increases. The fused multi-convolution feature has a higher recognition accuracy than a single convolution feature under the dataset, indicating that multi-feature fusion has strong robustness.

It can be seen that the information embedding features of edible mushroom samples obtained by the HMSE algorithm are better than the original information embedding features of edible mushroom samples in Figure 4, especially on the CONSE, SYNC, and EXEM models, the edible mushroom obtained by HMSE is better than the embedding feature of the information of the bacteria samples has greatly improved the recognition accuracy.

(7) $$\begin{array}{c} I\left(i,t-\frac{i}{n}\right)=ai\left(t\right)i\left(n-t\right)-bi\left(t-1\right)\left(\frac{1-n}{1-t}\right)-\left|t\left(n\right)-1\right|=0. \end{array}$$

For example, on the 2-hops test set, the top-5 recognition rate of HMSE combined with the CONSE model reaches 27.5%, which is 8.6% higher than the original edible fungus sample information embedding recognition rate. And on the whole, the recognition rate of HMSE in the above three models has been improved by nearly 1–2%. However, for the GCNZ and SGCN models, the information embedding of edible mushroom samples obtained by the HMSE algorithm has a weak overall improvement in the recognition rate.

(8) $$\begin{array}{c} \text{forerunner}\left(r,s\right)=\left[\begin{array}{cc} \text{max}\left(r+s\right) & \text{min}\left(r+s\right)\\ \text{min}\left(r-s\right) & \text{max}\left(r-s\right) \end{array}\right]. \end{array}$$

This is because GCNZ and SGCN are both models based on graph convolutional neural networks and WordNet hierarchical structure. In the process of model mapping, the hierarchical structure relationship of categories has been integrated, so the embedding effect of edible fungus sample information is obtained by the HMSE algorithm generally. In addition, when the convolution operation is performed in the category relationship graph, the eigenvalues embedded in the edible mushroom sample information will be continuously updated, which breaks the edible mushroom sample information obtained by the original HMSE algorithm. This just shows that the edible fungus sample information embedding obtained by the HMSE algorithm has better semantics and discrimination.

The initialization of Figure 5 is performed with a constant of 0.1. To further prevent overfitting, random deactivation with a neuron retention rate of 0.5 is used in the C51 layer of the basic classification network 1, the C102 layer of the basic classification network 2, and the C43 layer of the basic classification network 3, respectively. Each iteration randomly selects 25 samples from the training data as input, and the initial learning rate is set to 0.001, which is reduced to 0.9 of the current value after every 10 rounds of training. After 100 rounds of training, the recognition performance of the basic classification network is verified using test samples. The average recognition rates of the three basic classification networks reached 97.81%, 98.27%, and 97.57%, respectively. This result shows that the three networks have been effectively trained and can initially achieve accurate recognition of edible mushroom samples.

### 4.2. Small Sample Training of Toadstools and Edible Mushrooms

The auxiliary data set used by the pretraining model is selected from the ImageNet data set collected by the team through web crawling, manual annotation, etc. However, to achieve dimensionality reduction and speed up convergence in network training, the pooling operation is continuously used, and some parts are lost as the network deepens so that the diversity and distinguishability of the feature information of the “isomorphic” target task are not fully mined. The entire data set consists of 61 categories (by “species-disease-degree” points), 27 different degrees of disease image composition, the number corresponding to each class is shown on paper, and divided into 10 sub data sets, each sub data contains a picture of a species, including the health class and all disease classes, and then divide each data set randomly: 70% as the training set and 20% as the validation set, 10% as the test set.

(9) $$\begin{array}{c} \left\{\begin{array}{c} x\left(s\right)=\frac{u\left(s\right)\Delta u}{\Delta u^{\prime }\left(s\right)-s\left(t\right)},\\ y\left(s\right)=\frac{\Delta u\left(s\right)-\Delta u^{\prime }\left(s\right)}{\Delta s\left(t\right)-1}. \end{array}\right) \end{array}$$

Different category diagrams contain different constraints between categories. According to different category relationship graphs, each node will use different adjacent node features to update its features, so different category relationship graphs can extract different features for each node. The main function of the multi-scale graph convolution module is to increase the diversity of features in the width of the network, thereby improving the generalization ability of the models in Table 2.

The use of the standard cross-entropy function and the use of the focal loss function are compared from the two aspects of accuracy and loss value, where ResNet50_F represents the ResNet50 network with the Focal loss function, and ResNet50_S represents the ResNet50 network with the cross-entropy loss function. The model using the focal loss function achieves a recognition rate of 95.31% in the classification of crop leaves. Compared with the model using the standard cross-entropy function, the classification accuracy has not improved much, but the test loss value has dropped a lot. Using the test loss value of the standard cross-entropy function model is about 0.13, while the test loss value of the model using the focal loss function is only about 0.07.

### 4.3. Small-Sample Integration of Heterogeneous Edible Tannin

According to the small sample analysis of 4 deep heterogeneous edible mushrooms, the recognition accuracy of VGG-16NET and improved VGG is higher than that of AlexNET and ResNet-50, because VGG-16NET and improved VGG pass the combination and stacking of 3×3 filters, to extract the rich and small features in the disease area of the poisonous crops. Therefore, the recognition effect of AlexNET and ResNet-50 is worse than that of VGG-16NET and improved VGG. At the same time, the improved VGG network adjusts and optimizes the network structure to make the recognition accuracy rate higher than VGG16.

(10) $$\begin{array}{c} \text{sig mod}\left(\sum_{\Delta u}\Delta u-\Delta u^{\prime }\left(s\right)+b\left(\frac{\Delta u-s}{\Delta u^{\prime }\left(s\right)}\right)\right)=\sum \frac{\Delta u}{\Delta s}. \end{array}$$

Through the preprocessing operation, the samples can meet the input requirements of training the classification model, and the target task recognition error caused by the irregular data set and other problems can be reduced. Different from the ResNet model, which directly adds and fuses the network features of the previous layer with the network features of the latter layer, the dense connection mechanism splices and fuses the output features of all the previous layers and uses it as the input of the current layer network in Figure 6.

By using the Inception-v3 model and the transfer learning mechanism, the results of the two classifications of edible fungus samples and poisonous crop diseases are very stable and have high recognition accuracy. However, the recognition accuracy of the eight-classification task of edible fungus samples and toxin crop diseases is low, which indicates that Inception is difficult for the Inception-v3 model to identify the specific species of toadstools in various crop disease categories.

It can be seen from the figure that the MobileNet recognition model with different parameters can well complete the two-classification task of edible fungus samples and poisonous crop diseases. In the multi-classification task of poisonous crop diseases, the accuracy is much lower than in the two-classification task. In addition, the parameters of MobileNet will also have an impact on the identification rate of plant diseases. When the size of the convolution kernel and the input image are larger, the classification accuracy is higher, but it will occupy larger storage space and affect the recognition speed.

## 5. Application and Analysis of a Small Sample Recognition Model for Toxins and Edible Mushrooms Based on Graph Convolutional Neural Network

### 5.1. Graph Convolutional Network Data Preprocessing

In the segmentation part, the image in the input software is segmented using the improved graph convolutional network data to obtain an image containing only lesions, and the images containing only lesions are input to the next recognition part for recognition; in the recognition part, using the improved VGG network to identify the segmented images. The system mainly consists of two modules: front-end focusing index, which extracts potential target areas from large and wide edible mushroom sample images and generates a series of initial assumptions about target type, structure, posture, and other information, and realizes the extraction and coarsening of target slices. Classification: back-end iterative classification, complete target feature prediction, extraction and matching, and revising front-end assumptions.

(11) $$\begin{array}{c} \frac{\text{log}\left(m,n\right)}{\Delta m-1}-\frac{\text{log}\left(m,n\right)}{\Delta n-1}-\frac{\text{log}\left(m,n\right)}{\Delta m\Delta n}=\sum \frac{\text{log}\left(m,n\right)}{\Delta m\Delta n-1}-1. \end{array}$$

It can be seen that the initial training accuracy and validation accuracy of the VGG network framework are higher than those of the other three networks, similar to the data set of poisonous crop diseases. Among them, the training starting point and verification starting point of the Inception-v3 network are the lowest, but the accuracy of the final stable convergence is relatively high.

(12) $$\begin{array}{c} \frac{\text{exp}\left(f\left(a,b\right)-f\left(a\right)f\left(b\right)\right)}{\exp\left(\Delta f\left(a,b\right)-1\right)}\overset{\Delta n-1}{⟶}1-\text{exp}\left(\Delta a\left(\Delta b-1\right)-1\right). \end{array}$$

This shows that in this network, the characteristics that can be transferred from the large data set are limited, but the network can accurately capture various characteristics of crop diseases after parameter adjustment and re learning.

### 5.2. Simulation of Small Sample Identification of Toadstools and Edible Mushrooms

The selection comes from the experience accumulated by data mining researchers in their usual experiments. The researchers have limited experience and this process consumes resources. Second, the application range of artificially designed extractors is limited. For example, the sharpen operator can only be used for image sharpening. In the training process of the graph convolutional network, when the depth is too shallow, the higher-level and more comprehensive feature information of the plant cannot be captured, but when the depth is too deep, the increase of network parameters and the small data set will lead to overfitting. This leads to a decrease in verification accuracy. Therefore, depending on the size of the dataset and the difficulty of the recognition task, it is important to adjust the depth of the graph convolutional network in real-time and to compare the experimental results.

It can be seen that Inception in the single model of Figure 7. The Inception-v3 framework has the highest recognition accuracy for the edible fungus samples, which is 98.44%, and the VGG single frame has the worst recognition effect on crop diseases, with an accuracy rate of only 93.75%. In the multi-model ensemble experiment based on the direct average method, the ensemble model of DenseNet and Inception-v3, Inception. Integrated model of Inception-v3 and ResNet, DenseNet, Inception. The three model ensembles of Inception-v3 and ResNet all achieved the same highest validation accuracy of 99.22%. In the multi-model ensemble experiment based on the weighted method, the highest verification accuracy is 99.22%, which is comparable to the highest verification accuracy obtained by the direct average method. It can be seen that this result exceeds the highest accuracy rate of single-model recognition, indicating that the method based on graph convolutional network model ensemble can identify crop diseases based on single-mode.

### 5.3. Example Application and Analysis

Different adaptive learning rates are designed for different parameters for the small samples of poisonous and edible mushrooms. This method is easy to implement and has small memory requirements. It can continuously perform the weight update process of the graph convolutional network based on the training images of diseases and poisonous crop diseases until the optimal result is found to minimize the loss function. The learning rate is set to 0.001. Each of our experiments is run for 20 epochs, and within one epoch, all images in the training set are fully trained on the entire graph convolutional network. The optimization algorithm randomly selects a batch of samples in the training set to train the network. We set the batch sample size batch size to 64. Dropout is already mentioned in Figure 8, set it to 0.5. All experiments in this paper are implemented through the TensorFlow framework. TensorFlow uses data flow graphs for computation, and its workflow is relatively simple.

To test the generalization ability of the model, the crop identification model of edible sputum samples was applied to different datasets. The experimental results show that the recognition accuracy rate of multi-feature fusion on the dataset is generally improved, ranging from 1% to 10%, and the average recognition rate is about 91%.

(13) $$\begin{array}{c} 1-\frac{\sqrt{\text{exp}\left(f\left(a,b\right)-f\left(a\right)f\left(b\right)\right)}}{\text{exp}\left(a,b\right)}=\frac{\text{exp}\left(a+b\right)}{1-\text{exp}\left(a\right)\text{exp}\left(b\right)}. \end{array}$$

Among them, the correct recognition rate of the “isomorphic” type of toxin crop disease images has improved significantly, and the improvement is most obvious in the dataset, and the recognition accuracy has increased by about 10%. From the analysis of the recognition accuracy of the above six single diseases, it can be found that there are three diseases with relatively small values of recognition accuracy. These diseases are very similar in the shape, size, and texture of the lesions, and misjudgment often occurs; through the analysis of the data in the above table, it can be found that there are two data with larger identification accuracy, specifically verticillium wilt 96.08%, and 97.48% of leaf blight. The specific reasons for the high identification accuracy of the two diseases were analyzed, and it was found that this was caused by the obvious performance of the veins and leaf edges after the leaves were diseased.

But as the network depth increases, using transfer learning on the small dataset in Figure 9 gradually outperforms training from scratch. This is because the network with 3 or 4 convolutional layers can learn limited features and cannot learn more extensive visual features from the PlantVillage dataset to fit on the cucumber and rice disease datasets. When the network reaches a certain depth, the initial classification accuracy obtained using transfer learning is significantly higher.

(14) $$\begin{array}{c} \left\{\begin{array}{c} \sum p\left(a,b\right)-p\left(a\right)p\left(b\right)=1,\\ \frac{\text{exp}\left(\text{sig}\left(a,b\right)\right)}{\text{sig}\left(1-f\left(a\right)f\left(b\right)\right)}=1. \end{array}\right) \end{array}$$

In the case of training from scratch, as the depth of the network increases, the graph convolutional network has serious overfitting problems on the small-sample datasets of cucumber and rice disease edible mushrooms. Generally, fewer network layers cannot learn enough features to identify disease types, and more network layers will lead to overfitting on small datasets.

(15) $$\begin{array}{c} w\left(h\left(x\right)<1\left\|\right)h\left(x\right)-h\left(x-1\right)<1\right)=\frac{\sum p\left(a,b\right)-p\left(a\right)p\left(b\right)}{\sum p\left(a,b\right)-p\left(a\right)\sum p\left(a,1\right)-p\left(a\right)\sum p\left(a,b\right)-ap\left(b\right)}. \end{array}$$

Given the problem that the recognition rate of target tasks is not high due to the existence of fine-grained image data samples, the multi-layer convolution features in the network structure are fused to replace the feature output of the last convolution layer.

The larger the dataset is, the more information and distribution patterns the network can capture. As can be seen for our cucumber and rice disease datasets, when the network reaches a certain depth, transferring with a pretrained model obtained from the PlantVillage dataset can achieve higher accuracy than training from scratch. Our dataset background is more complex than the PlantVillage dataset. Furthermore, the sample distribution of each disease in our dataset is not uniform. Better transfer results can be obtained if we reduce the complexity of the background and make the number of samples per class uniform.

Since the scale of the PlantVillage dataset is larger than our dataset, the pretrained model in Figure 10 can achieve relatively high disease identification accuracy, which indicates that the scale of the training dataset has a great impact on the network's identification results. The most obvious is that on a graph convolutional network with 8 convolutional layers, using transfer learning, the identification accuracy of the disease dataset can be improved by 7.59% compared with the de novo training of the network. Using transfer learning to tune the parameters of the PlantVillage pretrained model on a network with 5 convolutional layers, our dataset can achieve a classification accuracy of 90.84%.

## 6. Conclusion

Aiming at the problem of the decline of the network recognition ability under the small sample of edible tannin, this paper studies the method of fine-tuning the target recognition method of edible tannin samples by a convolutional neural network. Using the parameters of the source domain pretraining model to initialize the network can alleviate the low generalization ability of the network caused by insufficient training samples, effectively improve the training efficiency and target recognition ability of the network, and solve the problem of deep graph convolution network model and parameter fine-tuning strategy recognition. The MobileNet network with different parameters is used as the underlying feature extractor for feature extraction, and then the classification model is used to identify the poisonous crop disease and the poisonous crop disease. Based on this theory, we have developed the identification system of plant diseases based on the MobileNet model and the Inception. The Inception-v3 model of the plant disease identification system of the toadstools. The easiest way to fuse feature maps of different depths is to directly concatenate all feature matrices to build a feature dictionary, and then input the classification layer for training. This operation will use each feature map in turn, because different feature maps contain extremely high similarity features, or some features have little impact on the recognition results, direct use will not improve the efficiency and increase the computational overhead. Therefore, before feature concatenation, to remove redundant information and reduce computational overhead, a necessary operation is to perform dimensionality reduction processing on each feature matrix.

## Figures and Tables

**Figure 1:** Graph convolutional network solution data evaluation.

**Figure 2:** Unilateral inhibition of diseased area.

**Figure 3:** Cascaded equivalent small sample overfitting distribution.

**Figure 4:** Graph convolutional network depth iteration information.

**Figure 5:** The distribution of information embedding features of edible mushroom samples.

**Figure 6:** Network feature addition fusion topology.

**Figure 7:** Fine classification of small samples of edible tannin.

**Figure 8:** Small sample adaptive learning rate of poisonous and edible mushrooms.

**Figure 9:** Graph convolutional network multi-feature fusion distribution.

**Figure 10:** Distribution of initial classification accuracy of graph convolutional network.

**Table 1:** Graph convolutional network solution set description.

Convolutional network node	Set ratio	Case a sample	Training samples	Inductive prediction
Vgg-1	0.30	3 × 3	Edible mushroom	10.82
Vgg-2	0.41	5 × 5	Azimuth angle	22.79
Vgg-3	0.67	9 × 9	Ground objects	27.41
Vgg-4	0.43	7 × 7	Scattering characteristics	18.31
Vgg-5	0.22	3 × 3	Azimuth angle	32.28

**Table 2:** Graph convolutional network category relationship.

Graph convolutional network case	Category relationship description
Functions are *p*(*a*, *b*) compared	For r, bar in zip (data, bar):
Use of the standard Δ*m*Δ*n*	Bar = ax1.bar (theta, data, alpha = 0.5)
Loss value Δ*n* − 1	Plt.figure (figsize=(8, 4))
From the two exp(*a*)	Ax1 = plt.subplot (111, projection = ‘polar')
And the use of exp(sig(*a*, *b*))	Ax1.set_title (‘spot fish')
Aspects of accuracy	Ax1.set_rlim (0, 12)
The focal loss Δ*m* − 1	*X* = np.linspace (0, 8*∗*np.pi, n)
Cross-entropy function *h*(*x* − 1) < 1	Sin_y = np.sin(x)
exp(*f*(*a*, *b*) − *f*(*a*)*f*(*b*))	Cos_y = np.cos(x/2)/2

## Data Availability

The data can be provided based on the request from the corresponding author.
